The article "Empirical Study on the Relationship between Agricultural Economic Structure Growth and Environmental Pollution Based on Time-Varying Parameter Vector Autoregressive Model" was retracted in 2023. Reasons: signs of a paper mill; suspected computer-generated content; unreliable results or conclusions; concerns about the data.

# Empirical Study on the Relationship between Agricultural Economic Structure Growth and Environmental Pollution Based on Time-Varying Parameter Vector Autoregressive Model

**DOI:** 10.1155/2022/5684178

**Published:** 2022-08-10

**Authors:** Xiaozhong Li, Feng Huang

**Affiliations:** ^1^Academy of Green Food Science of Heilongjiang, Northeast Agricultural University, Harbin, Heilongjiang 150030, China; ^2^College of Economics and Management, Northeast Agricultural University, Harbin, Heilongjiang 150030, China

## Abstract

In order to better demonstrate the relationship between agricultural economic structure growth and environmental pollution, an autoregressive model based on time-varying parameter vector was proposed. In the process of developing the research, this paper introduces the LDMI method, based on the time-varying parameter vector autoregression model, with the help of sampling formula calculation and other methods. Efforts were made to obtain credible conclusions. The experiment result shows that in this study, a total of 10,000 samples were taken. According to this value, 10000/116.15 = 86, which means that at least 86 unrelated samples can be obtained. Therefore, we can determine that each indicator mentioned in this paper has valid samples when it is introduced into the time-varying parameter vector autoregression (TVP-VAR) model for parameter estimation. After sampling detection image analysis and data calculation, the effect of energy structure, energy intensity industrial structure, and scale effect on the emission scale of environmental pollutants was obtained. It is proved that through the research of this paper, two main conclusions are finally obtained, and the influence of the five factors mentioned above is summarized.

## 1. Introduction

At present, in the process of their own continuous development, all countries in the world have invested more and more attention and strength in the work of ecological environment protection [1]. In terms of the actual situation in China, the scale of environmental investment has shown a steady and rapid growth, but at the same time problems such as ecosystem degradation and serious environmental pollution always exist. It is difficult to achieve a harmonious development between environment, resources, and economic development, and the contradiction between the two is increasingly prominent. Based on the perspective of China's industrial development, since the 1980s, up to now, the growth rate of industrial wastewater discharge has shown a relatively low degree of decline [2]. However, in addition, the discharge of industrial solid pollutants and industrial waste gas both showed an increase, with an average increase of 6.36% and 8.49% per year, respectively. China's efforts to clean up its environment have produced a paradox: the more polluted it is, the more polluted it is. As we all know, economic growth is the result of multiple influences. Since the reform and opening up more than 40 years ago, China's traditional economic growth mode has achieved relatively rich material wealth. However, it also consumes a relatively large scale of energy and resources, and also causes serious deterioration of the natural environment, which is bound to negatively impact its efforts to truly achieve sustainable economic growth. As the primary industry in China's national economic structure, the growth of agricultural economic structure should also invest more power in achieving the goal of improving the efficiency of resource utilization, so as to completely break the old development model [3].

The article "Empirical Study on the Relationship between Agricultural Economic Structure Growth and Environmental Pollution Based on Time-Varying Parameter Vector Autoregressive Model" was retracted in 2023. Reasons: signs of a paper mill; suspected computer-generated content; unreliable results or conclusions; concerns about the data.

Based on the actual situation of the current worldwide research on this issue, Dsmt4 Mean Divisia Index (LMDI) is used to decompose the specific degree of environmental pollution affected by economic growth, industrial structure energy consumption, and technological progress. Explore the basic factors that cause the change of environmental pollution in China, and describe the impact of each factor on China's environmental pollution in reality [4]. On this premise, the Time Varying Parameter Vector Auto Regression (TVP-VAR) model was used to analyze the Time evolution mechanism and influence channels of various variables on environmental pollution under the impact of differentiated lead Time. At the same time, the similarities and differences of each influencing factor on the mechanism of environmental pollution under the impact of different time points are investigated, so as to identify the positive factors that promote the reduction of pollution degree. In addition, the periodical characteristics of China's environmental pollution have been fully grasped and effective strategies to reduce environmental pollution levels have been explored [5].

In essence, during the study of economic development, what should be done is to conduct a systematic and comprehensive analysis of the various effects between economic development and environmental pollution, rather than focusing on the impact of economic development on the ecological environment. At the same time, we should also reverse the impact of the aggravation of ecological environmental pollution on economic development. However, as far as the current situation is concerned, most Chinese scholars and experts only explore the relationship between the two aspects unilaterally [6]. In this case, there are obvious constraints and limitations in the generated conclusions, which cannot be effectively applied in the whole country. The applicability is often insufficient, and it is difficult to provide reference value for the economic development of most regions in China to realize circular economy. Because of this, in order to change this situation and further realize the establishment and improvement of theoretical basis, this paper will use more scientific methods to study the relationship between the growth of agricultural economic structure and environmental pollution [7].

The article "Empirical Study on the Relationship between Agricultural Economic Structure Growth and Environmental Pollution Based on Time-Varying Parameter Vector Autoregressive Model" was retracted in 2023. Reasons: signs of a paper mill; suspected computer-generated content; unreliable results or conclusions; concerns about the data.

## 2. Literature Review

No matter from the perspective of the research in China or other countries in the world, many experts and scholars explain the causes of environmental pollution changes. They usually start from four different perspectives, namely, economic growth, industrial structure, energy consumption, and technological progress. Deep integration of China's economic and social development with the above four causes can explain the change of environmental pollution level to a certain extent.

Based on the technology, most of the current worldwide studies can be regarded as forming a consensus, that is, it is generally believed that technological progress can reduce the emission of environmental pollutants by reducing the emission reduction cost. However, it has also been found that changes in the elasticity of substitution between the polluting technology sector and the clean technology sector can lead to the following situation: Environmental pollution will be affected by uncertainty from the level of technology if there is a large elasticity of substitution between the two sectors; if the elasticity of substitution between the above two sectors is small, then strong and relatively sustainable environmental policies are needed to effectively promote enterprises to focus on clean technologies. If the intensity of environmental regulation shows a downward trend, the frequency with which companies use polluting technologies is likely to increase. At present, relevant literature in China has pointed out that the elasticity of substitution between polluting technology sector and clean technology sector in China is too small. Under such circumstances, most enterprises tend to pay more attention to the improvement of polluting technology level in the process of development, that is, resource-consuming production technology level. In other words, enterprises do not pay enough attention to clean technology. In this case, there is a certain deviation in the direction of technological progress, which makes it difficult to reduce the emission scale of environmental pollutants fundamentally. If the current direction of technological progress is difficult to return to the right track, it will be difficult to achieve compatible development between environmental protection and economic development [8].

The article "Empirical Study on the Relationship between Agricultural Economic Structure Growth and Environmental Pollution Based on Time-Varying Parameter Vector Autoregressive Model" was retracted in 2023. Reasons: signs of a paper mill; suspected computer-generated content; unreliable results or conclusions; concerns about the data.

Based on the level of energy consumption, the consumption of energy and resources can bring a large scale of carbon dioxide (CO_2_), nitrogen dioxide (NO_2_), sulfur dioxide (SO_2_), and other harmful substances that can pollute the environment, and these substances are also the key elements of air pollution and pollutant emissions(Figure 1). From the actual situation of domestic and foreign researches at present, when analyzing the adverse effects of energy factors on the ecological environment, the two aspects of energy structure and energy intensity are the main research directions of most scholars. Some scholars have come to a conclusion that there is an obvious positive correlation between pollutant emission scale and energy intensity by means of index analysis, grey system theory, regression analysis, and other methods. Generally speaking, emission reduction effect can be more effective in the case of reduced energy intensity.

In addition, coal has long been the main type of energy in China's energy consumption structure, which is also a basic cause of environmental pollution. For the realization of environmental benefits, the transformation and upgrading of energy structure can have a positive impact, especially for the realization of carbon intensity target, and the change of energy structure can play a large contribution, accounting for 45%. However, some experts and scholars found that China's current achievements in optimizing energy consumption structure to achieve emission reduction targets are not obvious when using the computable general equilibrium model [9].

Based on the perspective of economic growth and industrial structure, experts and scholars in related fields around the world have reached relatively uniform conclusions on the impact of these two factors on ecological environmental pollution. Specifically, this conclusion can be expressed as follows: with the continuous deepening of industrialization and the continuous improvement of economic development level, environmental pollution will develop to a more serious situation. When the level of economic development reaches a higher level, the industrial structure will also undergo certain changes and adjustments under such a background. The industrial economy with high pollution level and high energy consumption will be transformed into an efficient economy, and the pollution level will be reduced. The efficient economy refers to the clean environmental protection industry and high-tech industry. For example, some Chinese experts and scholars tend to focus on the obvious differences between China's regional economic development when studying this issue. When studying the relationship between environmental pollutant emission and economic development level in central and western China, it can be found that economic growth in eastern China has achieved the goal of effectively controlling environmental pollution at present. In the central and western regions, economic growth has led to an increase in pollutant emissions. It can be seen that the relationship between economic development and environmental pollution is usually consistent with the characteristics of environmental Kuznets, that is to say, the level of economic development promotes an inverted *U*-shaped relationship between itself and environmental pollution by means of influencing the industrial structure.

The article "Empirical Study on the Relationship between Agricultural Economic Structure Growth and Environmental Pollution Based on Time-Varying Parameter Vector Autoregressive Model" was retracted in 2023. Reasons: signs of a paper mill; suspected computer-generated content; unreliable results or conclusions; concerns about the data.

Moreover, from the current worldwide research conclusions, this curve has a strong applicability in the industrialized period of developed countries and regions. In addition, some scholars and experts verified this curve with differentiated data and found that they could prove the existence of this curve based on theory. But at the same time, there are some special cases where the curve will take on an inverted *N*-shaped shape or some other shape. The reason for the difference in curve shape may be that the regional scope and time scale of economic development stages used are also different. If we want to further analyze the reasons, we need to analyze the specific driving factors that affect the pollution path. Among the various driving factors, it is generally believed that the economic industrial structure is the most important one. Some experts concluded that the inverted *U*-shaped curve is caused by different types of industries after studying different countries [10].

In the process of studying the relationship between the growth of agricultural economic structure and environmental pollution, the economic factors that can affect environmental pollution are decomposed by means of logarithmic mean Di index (LMDI) method. Based on the time-varying parameter vector autoregression (TVP-VAR) model, the dynamic impact characteristics of each economic factor on pollutant emissions at different lead times and time points were explored.

## 3. Method

### 3.1. Solutions to Research Problems

In this paper, the LDMI method is used to decompose the factors affecting environmental pollution, which is based on this content as follows:

First, construct the Kaya identity:

(1) $$\begin{array}{c} pl=\frac{pl}{peM}\cdot \frac{peM}{pe}\cdot \frac{pe}{gdpI}\cdot \frac{gdpI}{gdp}\cdot gdp. \end{array}$$

In Formula (1), *pl* refers to the amount of environmental pollution; *peM* represents the meaning of coal consumption, its unit is ten thousand tons of standard coal; *PE* refers to the total energy consumption, and its unit is also ten thousand tons of standard coal. *gdpI* refers to the industrial output value, and its unit is 100 million yuan; *gdp* means gross domestic product (GDP), and its unit is also 100 million yuan. (*pl*/*peM*) = *edc*, this content means environmental pollution emission coefficient, that is, the pollution emission generated by burning coal per unit quantity; (*peM*/*pe*) = *ccr*, this content represents the meaning of the energy structure; (*pe*/*gdpI*) = *ei*, the meaning of this content is energy intensity; (*gdpI*/*gdp*) = *indr*, this content represents the meaning of industrial structure. After simplifying Equation (1), the following equation can be obtained:

(2) $$\begin{array}{c} pl=edc\cdot ccr\cdot ei\cdot indr\cdot gdp. \end{array}$$

In LMDI decomposition theory, there are two decomposition methods, namely, multiplication and addition, which can realize mutual transformation. In the calculation of the contribution of each variable, only one of them is needed to ensure the generality of the calculation results. In this paper, the additive decomposition method is used in the calculation [11]. The change in environmental pollution emission can be expressed as *pl*_*i*_ for phase I and PLI-1 for phase *i* − 1: **Δpl**_**i**_ **=** **pl**_**i**_ − **pl**_**i−1**_.

The article "Empirical Study on the Relationship between Agricultural Economic Structure Growth and Environmental Pollution Based on Time-Varying Parameter Vector Autoregressive Model" was retracted in 2023. Reasons: signs of a paper mill; suspected computer-generated content; unreliable results or conclusions; concerns about the data.

The environmental pollution emission coefficient effect, energy structure effect, energy intensity effect, industrial structure effect, and economic scale effect of phase i are expressed as Δ*pl*^*i*^_*edc*_, Δ*pl*^*i*^_*ccr*_, Δ*pl*^*i*^_*ei*_, Δ*pl*^*i*^_*indr*_, Δ*pl*^*i*^_*gdp*_. When the effect of each factor is measured year by year, the effect of each factor can be expressed by using the following equation:

(3) $$\begin{array}{c} \Delta pl_{e\;dc}^{i}=L\left(pl_{i};pl_{i-1}\right)\cdot \ln\left(\frac{edci}{edci-1}\right),\\ \Delta pl_{ccr}^{i}=L\left(pl_{i};pl_{i-1}\right)\cdot \ln\left(\frac{ccri}{ccri-1}\right),\\ \Delta pl_{ei}^{i}=L\left(pl_{i};pl_{i-1}\right)\cdot \ln\left(\frac{eii}{eii-1}\right),\\ \Delta pl_{indr}^{i}=L\left(pl_{i};pl_{i-1}\right)\cdot \;\ln\left(\frac{indri}{indri-1}\right),\\ \Delta pl_{gdp}^{i}=L\left(pl_{i};pl_{i-1}\right)\cdot \ln\left(\frac{gdpi}{gdpi-1}\right). \end{array}$$

The sum of the effects of the above five factors is the total effect, which is expressed by the following equation:

(4) $$\begin{array}{c} \Delta pl_{i}=pl_{i}-pl_{i-1}=\Delta pl_{edc}^{i}+\Delta pl_{ccr}^{i}+\Delta pl_{ei}^{i}+\Delta pl_{indr}^{i}+\Delta pl_{gdp}^{i},\text{ and}\\ L\left(pl_{i};pl_{i-1}\right)=\left\{\begin{array}{c} \frac{pli-pli-1}{\ln\left(pli\right)-\ln\left(pli-1\right)},\\ pli\text{ or }\left(pli-1\right),\;pli=pli-1, \end{array}\right.\;pli\neq pli-1,\;i=1981,1982,1983\ldots 2013. \end{array}$$

To sum up, five factors influencing the change of environmental pollution emission are decomposed by means of this method because the change rate of environmental pollution emission coefficient is relatively small. Therefore, another factor can be selected to replace this variable. According to the research of relevant scholars, this paper uses the representative variable of technology, capital productivity (*cp*_*i*_), as a substitute variable, and names this variable as technology effect.

The article "Empirical Study on the Relationship between Agricultural Economic Structure Growth and Environmental Pollution Based on Time-Varying Parameter Vector Autoregressive Model" was retracted in 2023. Reasons: signs of a paper mill; suspected computer-generated content; unreliable results or conclusions; concerns about the data.

### 3.2. Experimental Methods to Verify the Scheme

#### 3.2.1. Data Source Index Selection

Since the reform and opening up, China's economy has shown a trend of sustained and rapid growth. At the same time, China's rapid growth has provided a driving force for the development of the world economy and reshaped the world economic pattern. In order to further grasp the relationship between environmental pollution and industrial structure change and economic growth mode since China's reform and opening up, this paper selects 34 years' time series data from 1980 to 2013 as research data, and *The Compilation of 65 years' Statistical Data of New China* is the main source of data in this paper. Specifically, variable selection and data explanation mainly include the following five aspects [12].

*(1) Environmental Pollution Emission*. Environmental pollution discharge substances refer to the substances discharged from production activities that cause pollution to the ecological environment, including waste water, waste gas, and solid wastes. Based on the current accounting methods of pollution emissions in relevant literature around the world as a reference, three indicators of waste water (*Q*_1,i_) waste gas (*Q*_2,i_), and solid waste (*Q*_3,i_) are selected. In this, the unit of waste water is ten thousand tons, the unit of waste gas is one billion m^3^, and the unit of solid waste is also ten thousand tons. After completing the selection of the three indicators, they should be linearly standardized, respectively, so that the problem of nonsummation caused by different dimensions can be effectively solved [13]. The relevant data of the above three indicators studied in this paper mainly come from the *China Environmental Statistical Yearbook*, *China Environmental Yearbook*, and the *Statistical Data Compilation of New China in 65 Years*. The standardized formula used in calculation is as follows:

(5) $$\begin{array}{c} Q{∼}_{n,i}=\frac{Qn,i-\min\left(Qn,i\right)}{\max\left(Qn,i\right)-\min\left(Qn,i\right)}. \end{array}$$

In Formula (5), Max (*Q*_*n, i*_) and min(*Q*_*n*, *i*_) represent the maximum and minimum values of the NTH indicator in all years; *n* refers to pollution variables. Since there are only three indicators selected in this paper, *n* = 1,2,3; *I* represents the year. According to the relevant content mentioned above, *i* = 1981,1982,1983, 2013.

The article "Empirical Study on the Relationship between Agricultural Economic Structure Growth and Environmental Pollution Based on Time-Varying Parameter Vector Autoregressive Model" was retracted in 2023. Reasons: signs of a paper mill; suspected computer-generated content; unreliable results or conclusions; concerns about the data.

Similar to other research results, this paper also uses the equal-weight sum-average method to add the three indicators Q∼_1,i_Q∼_2,i_Q∼_3,*i*_ after linear standardization, and the result is used to represent the total amount of pollution emission, which is denoted as *pl*_*i*_.

*(2) Technical Effect*. The output brought by unit capital is recorded as the specific meaning of capital productivity variable, which is not only an important form that can represent the technical level but also has a close relationship with the value of pollution emission coefficient, and can directly reflect economic imbalance, overcapacity, and excessive investment. For example, when the value of capital productivity is small, the degree of environmental pollution will gradually deepen under the influence of excessive energy consumption and high capital waste. After leveling the capital variable (unit hundred million yuan) and the nominal GDP variable (unit hundred million yuan), respectively, and after effectively removing the price factor, real capital (RK_*i*_) and real output (RGDP_*i*_) can be obtained [14]. The variable of capital productivity can be expressed by the ratio generated by these two items, and it can also be used as the expression method of technical effect, which is *cp*_*i*_.

(6) $$\begin{array}{c} cp_{i}=\frac{{\text{RGDP}}_{i}}{{\text{RK}}_{\text{i}}}\text{.} \end{array}$$

*(3) Energy Factor*. As for pollutant discharge, energy consumption is one of the main ways to cause it. Based on the perspective of energy structure, nonrenewable and nonclean energy such as fossil energy still plays a very important role in China's current energy consumption structure. This situation is also a central factor in China's growing ecological pollution problem, which is influenced by the energy mix. In the research process, the representative variable of energy structure used in this paper is the proportion of coal in China's total energy consumption, which is represented by *ccr*_*i*_.

Based on the perspective of energy intensity, this paper collected relevant data of total energy consumption and expressed it with EN_*i*_. The GDP of each year from 1981 to 2013 was calculated with 1980 as constant price, namely, RGDP_*i*_.

The article "Empirical Study on the Relationship between Agricultural Economic Structure Growth and Environmental Pollution Based on Time-Varying Parameter Vector Autoregressive Model" was retracted in 2023. Reasons: signs of a paper mill; suspected computer-generated content; unreliable results or conclusions; concerns about the data.

After comparing the total energy consumption with it, the energy scale consumed per unit GDP can be obtained. The unit is ten thousand tons of standard coal, and this ratio is used to represent the energy intensity, expressed by means of EII. The formula is as follows:

(7) $$\begin{array}{c} ei_{i}=\frac{{\text{EN}}_{i}}{{\text{RGDP}}_{i}}. \end{array}$$

*(4) Structure Effect*. For thousands of years of China's development, agriculture has always played an important role in the development of China's national economy. The agricultural production period will consume a certain amount of energy but also cause the discharge of pollutants. Therefore, as the primary industry of agriculture, its proportion in China's industrial structure will lead to more and more pollution. In the process of improving China's industrial structure and changing its economic growth model, the emission of pollution may be alleviated to some extent. The proportion of the added value of this industry in the GROSS national economic product (GDP) is taken as the industrial structure variable and represented by indr_*i*_.

*(5) Scale Effect*. As China's economic development level and speed continue to accelerate and expand the scale of economic development, more and more abundant economic activities also lead to more pollutant emissions. Based on this background, when studying environmental pollution, it is usually necessary to introduce the real GDP variable into the scale effect as a key variable. At the same time, it is also possible to more effectively and intuitively reflect the specific changes in pollution emissions at the stage of differentiated economic development [15]. As mentioned above, after calculating the real GDP(RGDP_i_) of each year from 1980 to 2013, the logarithm of the obtained value was taken, and the logarithm was used as a specific variable representing different stages of economic development and scale effect, which was expressed by MEANS of lngdp_*i*_.

#### 3.2.2. Variation Characteristics and Influencing Factors of Environmental Pollutants

Figure 2 shows the variation characteristics of China's environmental pollutant emissions from 1980 to 2013. It can be seen from the figure that China's environmental pollutant emissions reached the maximum value in 1988 and the minimum value in 1997. In 2008, a serious economic crisis broke out worldwide. Under the influence of this event, the emission scale of environmental pollutants decreased to a certain extent. Based on this situation, this paper will take these years as time nodes when conducting research, and divide the period from 1980 to 2013 into four stages. Specifically, they are phase I (1980–1988), phase II (1989–1997), Phase III (1998–2008), Phase IV (2009–2013). Based on THE LDMI method, the contribution rate of each factor to environmental pollution in these four stages and the cumulative impact of each factor on environmental pollution are calculated. The results obtained are shown in Figure 3 and Table 1, respectively [16].

The article "Empirical Study on the Relationship between Agricultural Economic Structure Growth and Environmental Pollution Based on Time-Varying Parameter Vector Autoregressive Model" was retracted in 2023. Reasons: signs of a paper mill; suspected computer-generated content; unreliable results or conclusions; concerns about the data.

As can be seen from Figure 3 and Table 1, China is in the early stage of rapid economic development. Therefore, the intensity and attention invested in production technology are much higher than environmental protection technology. In addition, people have not formed a broad awareness of environmental protection in these two stages, resulting in the discharge of environmental pollutants which is not much affected by technology. In the subsequent development process of the third and fourth stages, as China invested more and more efforts in environmental regulation and cleaner production standards, the improvement of environmental protection technology promoted the development of production technology, and the technological effect was more effectively played. After studying the data, it can be found that the rationalization of energy structure can reduce the discharge scale of environmental pollutants to a large extent and relieve the environmental pressure more effectively. In addition, in the process of China's continuous development, the significant improvement of energy efficiency is an important measure to change the phenomenon of serious damage to the ecological environment, and also the key to energy conservation. At the same time, in the use of the LDMI method for environmental pollution factors of calculation, we can also come to a conclusion, namely, the optimization of industrial structure to the implementation of environmental mitigation effect provides strong impetus. In addition, we also should abandon the GDP theory; it encouraged scale effect to further promote the deterioration of the environment pollution. From the above-mentioned library environment kuznets curve theory, it can be found that the pollution of the environment will be affected by the economic development, while the existing only GDP theory will make local governments to overlook the sustainable development regardless of region capacity and environmental carrying capacity, leading to excessive development and more serious environmental pollution [17].

## 4. Experimental Result

The lag order of the model should be defined in advance before estimating the parameters by using the tVP-VAR model. In this paper, SC and AIC information criteria were used for judgment, and a time-varying parameter vector autoregression model with 1-order lag was determined [18]. 10,000 sampling times were completed by using the MCMC method, and corresponding parameter estimation results were finally obtained, as shown in Table 2.

The article "Empirical Study on the Relationship between Agricultural Economic Structure Growth and Environmental Pollution Based on Time-Varying Parameter Vector Autoregressive Model" was retracted in 2023. Reasons: signs of a paper mill; suspected computer-generated content; unreliable results or conclusions; concerns about the data.

As can be seen from the data in Table 2, all values of Geweke convergence diagnostic value (CD) do not exceed 1, which means that this content does not have a significance level and does not reach the 5% critical value of 1.96. Based on this situation, we can determine as follows: the null hypothesis converging to a posterior distribution cannot be rejected, and the sample finally converges. In addition, it can be seen from Table 2 that the value of noneffective factors has not reached a high level, and the item with the largest value is only 116.15. A total of 10,000 samples were taken in this study. According to this value, 10000/116.15 = 86, that is to say, at least 86 unrelated samples can be obtained [19]. Therefore, we can determine that each indicator mentioned in this paper has valid samples when it is introduced into the time-varying parameter vector autoregression (TVP-VAR) model for parameter estimation. The impulse response function of differential time point and differential lead time in the TVP-VAR model is shown in Figures 4–9.

From Figure 4(a) different time points and Figure 4(b) different lead periods, we can know that the emission scale of environmental pollutants can be reduced under the influence of technological effects.

According to the analysis of Figure 5(a) different time points, Figure 5(b) different lead times, and Figure 6, we can know that the discharge of environmental pollutants will be affected by the positive impact effect of energy structure.

According to Figure 7(a) different time points and Figure 7(b) different lead periods, it can be seen that the emission of environmental pollutants will be affected by the negative impact effect of energy intensity.

In Figure 8(a) different time points and Figure 8(b) different lead periods are studied, and a conclusion can be drawn that the emission scale of environmental pollution will be affected by differentiation from the industrial structure [20].

According to Figure 9(a) different time points and Figure 9(b) different lead times, it can be seen that there is a positive correlation between environmental pollution emissions and scale effect [21–24].

## 5. Conclusion

Through the discussion and research of this paper, with the aid of time-varying parameter vector autoregression model, the following two conclusions can be drawn for the relationship between the growth of agricultural economic structure and environmental pollution.

The article "Empirical Study on the Relationship between Agricultural Economic Structure Growth and Environmental Pollution Based on Time-Varying Parameter Vector Autoregressive Model" was retracted in 2023. Reasons: signs of a paper mill; suspected computer-generated content; unreliable results or conclusions; concerns about the data.

First, the impact effects of technological progress on the emission scale of environmental pollutants are all negative, and the productivity of enterprises and the cleanliness of products can be effectively improved under the background of the continuous development of green and environmental protection technologies, thus giving rise to the innovation compensation effect. At present, China has not really changed the irrational energy consumption structure, and the impact effects of different time points and lead times on the emission scale of environmental pollutants are all positive, and the time-varying characteristics are not obvious. In general, although the pollution effect caused by irrational energy structure is relatively clear, it will not last too long.

Second, the emission of environmental pollutants can be greatly reduced under the background of greatly improving energy efficiency. However, at the same time, the scale of pollutant emissions will also be affected by the rebound effect of energy intensity, and there are not enough positive factors that can exert internal constraints to promote emission reduction effect in China at present. The relationship between the degree of environmental pollution and industrial structure is getting closer and closer. The impact of scale effect on environmental pollution shows a strong characteristic of persistence.

## Figures and Tables

**Figure 1:** Agricultural environmental pollution.

**Figure 2:** Variation characteristics of environmental pollutant emissions in China from 1980 to 2013.

**Figure 3:** The contribution of various factors to environmental pollution changes.

**Figure 4:** Impulse response function of environmental pollution under technology shock. (a) Different time points. (b) Different lead times.

**Figure 5:** Impulse response function of environmental pollution under energy structure impact. (a) Different time point. (b) Different lead times.

**Figure 6:** The changing characteristics of China's energy structure during 1980–2013.

**Figure 7:** Impulse response function of environmental pollution under energy intensity shock. (a) Different time points. (b) Different lead times.

**Figure 8:** Impulse response function of environmental pollution under industrial structure impact. (a) Different time points. (b) Different lead times.

**Figure 9:** Impulse response function of environmental pollution under economic scale shocks. (a) Different time points. (b) Different lead times.

**Table 1:** The cumulative effect of each factor in four stages on the discharge of environmental pollutants during 1981–2013.

Time	Year	Technical effect	Energy structure	Energy intensity	Industrial structure	Scale effect
Phase I	1980–1988	0.3081	0.0396	−0.2994	−0.0577	0.0765
Phase II	1989–1997	0.4642	−0.0296	−0.2578	0.0350	0.0532
Phase III	1998–2008	−0.0720	0.0028	−0.2362	0.0292	0.0912
Phase IV	2009–2013	−0.4662	−0.1359	−0.3633	−0.1844	0.0791
All	1980–2013	0.2341	−0.1231	−1.1567	−0.1779	0.3000

The article "Empirical Study on the Relationship between Agricultural Economic Structure Growth and Environmental Pollution Based on Time-Varying Parameter Vector Autoregressive Model" was retracted in 2023. Reasons: signs of a paper mill; suspected computer-generated content; unreliable results or conclusions; concerns about the data.

**Table 2:** TVP-VAR model parameter sampling and estimation results.

Parameter	Mean	Standard deviation	95% lower confidence interval	95% upper limit of confidence interval	Geweke convergence diagnostic value (CD)	Noneffective factor
sb1	2.0896	1.5057	0.4952	6.2266	0.787	116.15
sb2	1.8556	1.1554	0.4910	4.9109	0.525	86.83
sb3	0.1500	0.4002	0.0419	0.5832	0.567	14.96
sb4	0.1276	0.3190	0.0419	0.4909	0.863	18.15
sb5	0.2416	0.1844	0.0562	0.7351	0.719	103.72
sb6	0.1836	0.1620	0.0517	0.5915	0.390	55.60

## Data Availability

The labeled dataset used to support the findings of this study are available from the corresponding author upon request.
